The article "Estimation of Parameters on Probability Density Function Using Enhanced GLUE Approach" was published in 2022. Journal: Comput Intell Neurosci.

# Estimation of Parameters on Probability Density Function Using Enhanced GLUE Approach

**DOI:** 10.1155/2022/3250499

**Published:** 2022-10-14

**Authors:** Fuad S. Alduais, Neveen Sayed-Ahmed

**Affiliations:** ^1^Department of Mathematics, College of Science and Humanities in Al-Kharj, Prince Sattam Bin Abdulaziz University, Al-Kharj 11942, Saudi Arabia; ^2^Statistics Department, Faculty of Commerce (Girl Branch), Al-Azhar University, Cairo, Egypt

## Abstract

The most essential process in statistical image and signal processing is the parameter estimation of probability density functions (PDFs). The estimation of the probability density functions is a contentious issue in the domains of artificial intelligence and machine learning. The study examines challenges related to estimating density functions from random variables. Based on minimal predictions regarding densities, the study discusses a framework for evaluating probability density functions. During the Bayesian approach, which is to generate correct samplings that reflect the probability aspect of the variables, sampling is widely used to estimate as well as define the probabilistic model of unknown variables. Because of its effectiveness and extensive application, the generalized likelihood uncertainty estimation (GLUE) method has earned the most popularity among the various methodologies. The Bayesian technique allows parameters of the model to be estimated using prior expertise in the parameter results and experimental observations. The study uses a number of engineering issues that were lately looked into to illustrate the effectiveness of the upgraded GLUE. As the focus is on the examination of sampling effectiveness in view of engineering components, only a brief summary is provided to describe every challenge. The suggested GLUE method's outcomes are contrasted with those obtained using MCMC. Nevertheless, using the GLUE approach, the model's mean squared error of prediction is substantially higher than that of the previous algorithms. The methods' results are affected by the assumptions being made on parameter values in advance. The concepts of prediction accuracy, as well as the utility of geometric testing, are presented. Such notions are valuable in demonstrating that the GLUE approach defines an inconsistent and incoherent statistical inference process.

## 1. Introduction

Parameter estimate is described as the method for the determination of estimates for parameters that govern the response of the structure, provided that the system architecture is established. Parameter estimation is a field of statistics that involves estimating the parameters of a distribution utilizing data samples. For precise predicted results as well as effective model-based decision criteria, complete model parameter estimation is essential. Basic knowledge depended on expert information and ideas obtained through experimentation are still the two forms of knowledge commonly accessible for calculating the parameters of certain models. Just the information is utilized to estimate parameters of the model throughout most statistical methods, including the least squares method [1]. Throughout several engineering challenges, including such analysis of structures at the designing phase or the health maintenance of existing systems, parameter estimation is always a necessary step. Material parameters of the constitutive equations that have a substantial impact on the reliability of the simulation analysis must be accurately determined using data from direct or indirect observations during the design phase. In order to determine the remaining useful capacity of structures, degradation parameters of the underlying physical concept in decaying frameworks must be estimated utilizing observed data throughout time.

The article "Estimation of Parameters on Probability Density Function Using Enhanced GLUE Approach" was published in 2022. Journal: Comput Intell Neurosci.

In contrast to conventional techniques, the Bayesian methodology enables the estimation of parameter estimation to include not only observations but also preconceived notions regarding parameter values. Those approaches also have the benefit of being able to analyze the effects of parametric uncertainties on simulated data. The unidentified model parameters were represented as a stochastic process with a probability distribution that indicates uncertainty regarding model parameters in the Bayesian network [2]. The probability is adapted from previous information regarding parameter values proceeding to gather additional data. If no knowledge is accessible, an uninformative preceding distribution can be defined. Several of the parameters in ecological models, however, are immediately relevant, and minimum and maximum ranges can typically be specified for these values. In these circumstances, the previous parameter distributions could be determined by a homogenous distribution, for example. Bayes' theorem determines the parameter distribution prior to data collection. The previous distributions and the data both influence the posterior parameter distributions. As a result, that distribution comprises all of the knowledge on the design variables that are presently available [3].

The posterior parameter distributions cannot be computed and analyzed owing to the difficulty of certain prototypes (nonlinearity, large number of parameters). Nevertheless, as machines get more powerful and newer methodologies emerge, the Bayesian approach becomes extra manageable, also for complicated techniques. In recent years, the Bayesian network is becoming popular as a method for quantifying the uncertainties of variables in estimate processes. The following is a summary of the Bayesian approach: create a posterior probability for the uncertain variables derived from empirical data that indicates the level of confidence. Generate sampling that reflects the parameter range [4]. The variables of a framework are not considered particularly to be characterizations of physically constructive amounts with true (albeit unknown) principles in the traditional Bayesian approach, but instead, provisional “fake” or “suitable” amounts of uncertainties (on that every uncertainty is predictable) to be marginalized out by using one's posterior probability density that is acquired from observational data through the Bayesian inference procedure. If the goal is “parameter estimation,” it is explicitly presumed that the variables have a true but uncertain value that could be approximated once the probability density was already computed, based on either the maximum probability value or the anticipated value [5].

The article "Estimation of Parameters on Probability Density Function Using Enhanced GLUE Approach" was published in 2022. Journal: Comput Intell Neurosci.

The probability density function (PDF) is a probability function that indicates the distribution of a continuous probability distribution that falls among a set of values. In other terms, the probability density function calculates the probability of discrete random variable values [6]. A probability distribution function or simply a probability function is another name for it. However, several other reports indicate the function as a function across a wide range of values. It is also known as the cumulative distribution function or the probability mass function (PMF). PDF (probability density function) is established for continuous random variables, while PMF (probability mass function) is established for discrete random variables [7]. The probability density function is specified as the average of the variable density distribution over a certain range. Letter *f* stands for it (*x*). At any point on the graph, the variable is positive or non-negative, as well as the integral, more precisely the defined intrinsic of PDF over the entire facility, is always one. The likelihood of the occurrences is usually shown by a bell curve on the graphs of PDFs.

A continuous random variable's probability density function (PDF) could be easily estimated using the notion of power spectral density (PSD) estimation. A PDF varies from a PSD in that it has a space constraint, whereas a PSD does not. In pattern classification, imaging, and signal processing, the estimation method of probability density functions (PDFs) is essential [8]. For the identification of the fundamental signals, several actual duration signal processing applications demand autonomous, steady, and statistically developed management. Generating parameter estimates in the foundation of simple image processing tasks, including recognition and classification, is a typical difficulty that is encountered when using statistical methodologies. The system variable's probability density function form could be used as a better analytical technique to fully model the performance of a stochastic process. As a result, for management strategy creation with diverse design criteria, a PDF-based approach delivers accuracy and flexibility [9]. In general, the posterior distribution is expressed as a sophisticated or explicit formulation in terms of the dimensions, making sample generation difficult and preventing the use of typical probabilities functional approaches. Throughout this approach, numerous systems have been employed.

The article "Estimation of Parameters on Probability Density Function Using Enhanced GLUE Approach" was published in 2022. Journal: Comput Intell Neurosci.

The generalized likelihood uncertainty estimation (GLUE) approach has recently been demonstrated as a statistically efficient method. Beven and Freer [10] proposed the generalized likelihood uncertainty estimating methodology based on notions that, while articulated in various terminologies, are quite comparable to Bayesian concepts. GLUE “represents the evolution of Bayesian or fuzzy averaging processes to the less formal likelihood or fuzzy measures,” as per the researcher. A notable part of the GLUE technique is the idea of “the fewer formalized likelihood,” which provides the fundamental point of variation through Bayesian inference. The GLUE approach is a Monte Carlo technique with the goal of identifying a variety of cognitive modeling from a range of model/parameter combinations. On the basis of various information and expertise, the phrase “behavioral” refers to concepts that are deemed “acceptable,” that is, not ruled out. To construct GLUE, a significant amount of iterations are carried out for a model output with various parametric configurations picked at random using preceding parameter distributions. Every set of model parameters is allocated a probability value, which is a statistic that measures in what way that specific variable grouping (or model) replicates the systems, by evaluating expected and observed responses. Greater likelihood functional numbers often propose a good match among predicted results as well as the clarifications. The complete collection of imitations is later divided into behavioral and nonbehavioral parameters depending on a cutoff threshold [11].

The idea behind this strategy is to discretize the number of variables by using the posterior probability to create a large number of model parameters. From the probability and probability density values, values are determined for each parameter value. Even though Beven [12] claim that GLUE has been created to address uncertainty related to several types of errors, including “error due to vaguely understood model parameters as well as input variables, and error associated with measurement techniques used during the calibration process, as well as error due to modeling process deficiency,” in actuality, it only accounts for them implicitly through the stochastic nature of the model residuals. In fact, GLUE is dependent on the structural model, inputs mistakes, and initial values, which would not be considered unpredictable [13]. With the underlying understanding of cumulative mistakes, unpredictability is only believed to be caused by an inadequate knowledge about modeling attribute values, as well as perhaps by forecast and observational errors. The technique utilizes Monte Carlo (MC) analyses in combination having Bayesian estimates and uncertainty propagating to translate the variability in the model development onto the dimensional space. The GLUE methodology rejects the idea of a single global optimum input parameter inside a structural model, rather than acknowledging the acceptance of distinct parameter values that are as good at delivering fit forecasting accuracy within a model structure. The analysis of different model parameters inside pseudo-Bayesian MC architecture specifically addresses the idea, known as equifinality. The GLUE process produces parameter distributions including related uncertainty boundaries that are dependent on the available observational data [11].

The article "Estimation of Parameters on Probability Density Function Using Enhanced GLUE Approach" was published in 2022. Journal: Comput Intell Neurosci.

The prevalence of GLUE could have been credited to its theoretical accessibility, comparative convenience of development and use, and capacity to control a variety of error models and theories without requiring large changes to the method itself. Although this advancement, GLUE has been criticized since it cannot be officially Bayesian in necessitating particular judgments on the likelihood function as well as cutoff threshold dividing behavioral and nonbehavioral techniques, and it will not be adopting a quantitatively reliable error method. Furthermore, in several of the GLUE implementations, a very simple MC sampling strategy is utilized to sample from the distributions of the prior parameters and identify a well-distributed variety of cognitive modeling including their corresponding prediction simulations uncertainty [14]. Practitioners of the GLUE technique typically use basic random selection or, in certain situations, the much more accurate Latin hypercube sampling (LHS) procedure to survey the prior parameter distributions. Despite their ease of implementation, random sampling techniques were uncertain to intensively illustrate the limited space close to the finest solution with a dense distribution of values. The hypothesis is that by utilizing an adaptive sampling technique that updates the search direction based on information from previous draws, significant gains in sampling can be made. Such a strategy would almost certainly result in more reliable parameters and prediction error estimations [15].

The article "Estimation of Parameters on Probability Density Function Using Enhanced GLUE Approach" was published in 2022. Journal: Comput Intell Neurosci.

Numerous engineering issues that have lately been researched are used to highlight the effectiveness of the GLUE. Only a brief summary of every issue is provided because the analysis of sampled effectiveness in perspective of engineering fields is the main topic. The suggested GLUE method's outcomes are contrasted with those from the MCMC. In every one of the challenges, the procedure is carried out with nl = 10,000 LHS and nm = 5000 MCMC iterations. Several approaches to solve this problem were published in the statistical literature; however, satisfactory solutions in actuality are uncommon in engineering applications. The marginal PDF of every variable from the joint posterior distribution is used as a proposal distribution throughout this work, which results in a more robust technique. Because the numerical solution is computationally costly when constructing the marginal PDF, Latin hypercube sampling (LHS) is used to generate the PDF in a discrete manner. The contribution of the study is to illustrate the efficiency of the suggested GLUE strategy; multiple engineering problems with unknown parameters are solved using a Bayesian approach. The article is divided into six sections. In Section 2, existing techniques are briefly discussed. The problem statement is discussed in Section 3.  Section 4 covers the GLUE approach, including the implementation of GLUE into PDF.  Section 5 contains the results and comments, as well as tables and graphs. Finally, the article is concluded in Section 6.

## 2. Related Works

The subject of combined Bayesian model evaluation and parameter estimation for sinusoids in white Gaussian noise is investigated in this study. The authors provide a unique Bayesian framework that provides us to construct a posterior distribution on the parameter space. That distribution is then used for everything in Bayesian statistics. However, a direct assessment of such a distribution as well as its properties, such as posterior model probability, necessitates the assessment of certain complex high-dimensional integrals. To execute the Bayesian computations, researchers design an efficient stochastic system based on reversible jumping Markov chain Monte Carlo techniques. The algorithm's convergence outcome is verified. The effectiveness of identification based on posterior modeling probability tends to exceed standard detection systems in simulations. Numerical approaches are required to evaluate such posterior distribution and its aspects of interest. To determine this posterior distribution, an affective computing optimization technique on reversible jumping MCMC techniques was developed. The outcomes of large simulated research reveal that modeling selection based on posterior model probability outperforms the other traditional criteria. Whenever dealing with scenarios with low SNR, limited sample sizes, or tightly packed frequencies, such a strategy is quite useful. Of course, computationally efficient approaches are a good option in more favorable scenarios. However, some approaches have significant flaws. First, because it might be huge, it is computationally expensive. Second, each parameter is assigned the same computing effort. In fact, several of the variables are irrelevant in practice since their posterior model probability is so low [16].

The article "Estimation of Parameters on Probability Density Function Using Enhanced GLUE Approach" was published in 2022. Journal: Comput Intell Neurosci.

Analyzing chemically interacting circulating currents with probability density function (PDF) approaches has many benefits. This brings an exceptional and practical solution to the closing issues that result through averaging or filtering the highly nonlinear chemicals' central component, as well as conditions that approximate other one-point physical phenomena (e.g., radiative emission) in the immediate continuity equation. The study is restricted to transportable PDF approaches, in which a formula dictates the development of the one-point, one-time PDF for a collection of factors that influence the localized thermochemical and/or hydrodynamic condition of a reacting system. PDF-based methodologies as subfilter-scale modeling techniques for large-eddy computation (filtered density function methods), PDF-based simulations of thermoelectric radiation heat transfer as well as turbulence–radiation interrelations, PDF-based features for soot and liquid fuel splatters, and Eulerian survey strategies for fixing simulated PDF analytical solution are among the significant developments mentioned. To underline crucial ideas, instances of applicability to canonical processes and laboratory-scale flames, including real combustion devices, are offered. Throughout the book, an endeavor has been made to achieve a balance between rigor and readability, covering depth and breadth, including essential science and actual implications. The analysis is required to respond to increasing the availability of PDF approaches and debunking common misconceptions regarding them. Although PDF approaches have generally been used to react to the ideal-gas combinations utilizing single-turbulence-scale simulations, knowledge from various mechanics and scales is easily included. However, because this technique cannot easily generalize to any three-dimensional geometrical layout, many PDF techniques have disregarded it [17].

The article "Estimation of Parameters on Probability Density Function Using Enhanced GLUE Approach" was published in 2022. Journal: Comput Intell Neurosci.

On the accelerating component, the probability distribution function has *R* = 690, which has provided observational evidence with probabilities fewer than 1007. That represents a significant improvement above previous observations, enabling us to assume that the fourth-moment convergence rate and the flattening are around 55. Researchers compared the probability distribution to that anticipated by numerous nonextensive statistically mechanics-inspired systems. They also discover that accelerator element stochastic models conditioning on a particle velocity with conditioning velocities up to 3 times the confidence interval are extremely non-Gaussian. The models based on log-normal statistical or multifractal analyses (Arimitsu) are quite comparable to the empirical pieces of evidence. Because the main distinction among the two models is the fundamental demographics (Tsallis or log-normal), the Tsallis stats assumption should be rejected in order to replicate the accelerated PDF's observable behavior. The appropriate reactive of the variable in the models to the diffusion equation and the use of log-normal statistical are in accordance with the improved Kolmogorov–Obukhov model of turbulent, which is recognized to capture well the properties of intermittent nature. The combined PDF of velocity and acceleration is likewise shown to be non-Gaussian. The velocity variability conditional on speed, on the other hand, is not consistent. Such findings have significant implications for the architecture of the stochastic equations necessary to simulate turbulent flow distribution [18].

Independent decision-makers' individuality is inextricably linked to group decision-making, therefore making attaining a group decision challenging. Several of the challenges is aggregating a small number of evaluations while accounting for individual identity or ambiguity using the probability theory. This tough problem is called probability distribution function aggregation (DFA). The study proposes a straightforward and effective solution to the DFA problem. The suggested approach's fundamental concept is to represent the DFA issue as a nonlinear system of a collection of probability distribution functions and to suggest a linear feedback iterative method to address the nonlinear model, resulting in a collective judgment or conclusion. A well-known DFA instance that was resolved using the Delphi method serves as an example of such a novel approach. The decision-making issue involves the DFA problem. As a result, the suggested technique is applicable to any decision-making task. The suggested terminology for methodically encoding the inaccurate group decision issue with the categorization of uncertainty into three forms, inadequate knowledge, ambiguous knowledge, and indeterminate details, would be another sign of this research. With the well-known Delphi technique, the recommended methodology was taken to a situation in the research. The method has been proved to be quite efficient; in the case of the example mentioned in this study, it took 3-4 iterations to attain convergence. The paper also came to the conclusion that the optimal aggregated dispersion functional must be limited and centralized. This discovery was used to create a system for calculating the starting weights in the suggested method. This broad notation is then applied to the specific DFA problem addressed in this study. DFA, on the other hand, has limited memory. It cannot hold any information of unlimited duration due to its finite memory [19].

The article "Estimation of Parameters on Probability Density Function Using Enhanced GLUE Approach" was published in 2022. Journal: Comput Intell Neurosci.

The analysis of signal obtained on a number of sensors to locate the position of the transmitter is adequate relevance that it has been handled under a variety of special case assumptions. In a noise/interference situation including an arbitrary covariance matrix, the main difficulty involves sensors with random positions including directing properties (gain/phase/polarization). The study is focused on two aspects of the problem: the many emitters component and the universality of the solution. The multiple signal classification (MUSIC) procedures are given, which also offer asymptotically accurate estimations of the following: (1) the percentage of event wavefronts existent; (2) instructions of the entrance (or emitter locations); (3) abilities and traverse correlation coefficients between many occurrence waveforms; and (4) noise/interference resilience. Instead of integration of an all-pole Fourier transform generated by white noise (i.e., autoregressive modeling, maximum entropy) or maximizing a probability underneath the premise that the vectors are zero average and Gaussian, MUSIC analyzes the information as the combination of specular reflection emission as well as noise (maximum likelihood for Gaussian data). Maximum likelihood minimizes a balanced aggregate of all component lengths, while MUSIC minimizes the length from the continuous to the signal subspace. There are demonstrations and correlations with maximum likelihood (ML) and maximal entropy (ME) approaches, as also traditional beamforming. Its application as a multiple frequency analyzer on data series is demonstrated. There are no assumptions concerning array geometry. The components can be placed in a regular or irregular manner, and their directed qualities (amplitude/phase) can change or be similar, as long as their polarization properties are all the same. The geometrical importance of certain vector space settings and the perception of a specific matrices eigenstructure, on the other hand, were overlooked [20].

The article "Estimation of Parameters on Probability Density Function Using Enhanced GLUE Approach" was published in 2022. Journal: Comput Intell Neurosci.

Automatic modulation recognition is beneficial for modulation schemes, software-defined wireless, and traditional wireless telecommunication networks. In this study, researchers look at how to detect the modulation scheme of a linear modulation index using a phase-based linear discriminant (ML) approach. Researchers suggest two approximation ML alternatives, which can provide close-to-optimal performances using minimized cost because the optimum ML technique is computationally expensive. Then, for segmentation and classification kinds of modulating configurations, researchers give a general performance assessment. Researchers develop a set of upper constraints on PCC that represent a trade-off between precision and calculation cost. Also addressed is the asymptotic behavior of phase-based ML classification techniques. Researchers have developed 2 approximation phase PDFs that are described as arithmetic operations, by using the Gauss–Legendre quadrature method and the semi-infinite Gauss–Hermite computation method. The initial stage PDF, on the other hand, has a unique feature. These two approximation phase PDFs produce a PCC that is unrecognizable from the ideal ones provided by the initialization step PDF, according to the simulation solution. To the extent that they would operate well for any SNR values of practical interest, these outperformed the Tikhonov PDF and the Fourier series technique. It is important to note that the semi-infinite Gauss–Hermite quadrature rule provides enough precision. However, at a low SNR, the Tikhonov PDF loses precision, and at a high SNR, the Fourier series technique loses accuracy. The Gauss–Legendre quadrature approximation gets less precise as well [21].

Regarding large-eddy modeling of turbulent spray combustible, a coherent probability density function (PDF)-oriented ignition modeling technique is established. In the form of limited frequency LES equations, a Lagrangian Monte Carlo technique for resolving the PDF numerical scheme is devised. An innovative pilot-stabilized ethanol spray flame is simulated using the LES/PDF technique. Droplet evaporation happens distant from the flame front in of this flame, resulting in the distance between the two operations. All across the duration of the flame, a high-temperature preflame region with a stratification combination is discovered. The flame front cannot propagate through all this evaporating but well-mixed fuel/air mixture due to the high fluid velocity of the droplet-laden air. When compared to investigations, there were significant differences in droplet inflow parameters. Droplet-turbulence interaction in the injecting pipe, in this instance, greatly alters inflow disturbance. For application with the LES technique, a continuous PDF methodology for turbulent spray ignition has been developed. In the framework of a low-Mach number LES solver, a Lagrangian Monte Carlo technique that faithfully regenerates the higher-order moments of the PDF was been created. An ethanol spray flame was studied using the LES/PDF method. The LES/PDF technique accurately replicated the results of the experiment. This was also discovered that an absence of data regarding the intake circumstances resulted in significant differences between simulation and experimental results. However, the PDF equations provided in that paper do not achieve the correct vector moment numerical scheme that is critical for continuity. Furthermore, because of the inherent unpredictability of the computations, using the transported-PDF technique in LES necessitates special numerical constraints [22].

The article "Estimation of Parameters on Probability Density Function Using Enhanced GLUE Approach" was published in 2022. Journal: Comput Intell Neurosci.

## 3. Problem Statement

The traditional parametric and nonparametric techniques for measuring density functions have a lot of shortcomings; parametric techniques generate poor results when dealing with unidentified distributions, whereas nonparametric methods necessitate a large number of construction measurements, storage capabilities, and computational power. As a result, the paper presented a method for assessing probability density functions since only minimal density estimates are given. Sampling is commonly used to estimate and describe the probabilistic model of unknown factors in the Bayesian approach, which is to provide accurate samplings that represent the probabilistic aspect of the parameters. The generalized likelihood uncertainty estimation (GLUE) approach has gained the most popular among the numerous methodologies due to its efficacy and wide application. The Bayesian method allows model parameters to be calculated based on prior knowledge of parameter outcomes and experimental measurements.

## 4. Proposed Methodology with Glue

### 4.1. Bayesian Technique

Bayesian theorem, the following equation provides the posterior parameter distribution [23]:

(1) $$\begin{array}{c} \left(\alpha |X\right)=\frac{\vartheta \left(X|\alpha \right)\vartheta \left(\alpha \right)}{\vartheta \left(X\right)}. \end{array}$$

Here, *X* is the measurements vector, *ϑ*(*α*) is the preceding parameter distribution, *ϑ*(*α|X*) is the posterior parameter distribution, *ϑ*(*X*) is a proportional variable given by the condition that the integration of *ϑ*(*α|X*)across the dimensional space approaches 1, and *ϑ*(*X|α*) is a probability function. Given the parameters, *ϑ*the probability is the value of the observation *X*. Its ratio is described by the inaccuracy probability distribution among modeled and measure actual data. It is clear that either the previous distribution or the emerged data have an impact on the posterior parameter distribution.

The article "Estimation of Parameters on Probability Density Function Using Enhanced GLUE Approach" was published in 2022. Journal: Comput Intell Neurosci.

### 4.2. Enhanced Generalized Likelihood Uncertainty Estimation

The work proposes an enhanced robust GLUE sample technique for multidimensional characteristics that provides proper sampling by using a marginal PDF as a proposed distribution. The summation of the targeted joint PDF with consideration of many other parameters excluding it defines the marginal PDF of any random variable. The GLUE approach works on the assumption that the posterior parameter distributions *ϑ*(*α|X*) may be approximated by a discrete probability distribution(*α*_*i*_, *r*_*i*_), where *r*_*i*_ is the likelihood connected with the parameter *α*_*i*_. The procedure is as follows [24, 25]:

(i) Construct *K* vectors *α*_*i*_, *i*=1,…, *K* at arbitrary out from preceding parameter distribution *ϑ*(*α*).
(ii) Compute the probability numbers *ϑ*(*X|α*_*i*_) and the probability density *ϑ*(*α*_*i*_), *i*=1, ..., *K*, related to the various parameter vectors created.
(iii) Compute
  (2) $$\begin{array}{c} \begin{array}{c} r_{i}=\frac{\vartheta \left(X|\alpha_{i}\right)\vartheta \left(\alpha_{i}\right)}{\sum_{j=1}^{K}\vartheta \left(X|\alpha_{j}\right)\vartheta \left(\alpha_{j}\right)},\\ j=1,\ldots ,K. \end{array} \end{array}$$
Where ∑_*i*=1_^*K*^*r*_*i*_=1.

The pairs (*α*_*i*_, *r*_*i*_), *i*=1,…, *K*, could be used to calculate different properties of the posterior distribution, such as the posterior means $\bar{\alpha }=\sum_{i=1}^{K}\alpha_{i},r_{i}$. The GLUE method implementation is simpler than the others because it only involves the specification of the overall variable of created parameter variables *K*.

The marginal PDF of a single variable *A* is parameterized as the total of the targeted combined PDF having regard to many other variables without it that is determined by

(3) $$\begin{array}{c} s\left(A_{i}\right)=\int^{}r\left(A_{1}\ldots A_{i-1},A_{i},A_{i+1\ldots .}A_{n}\right)fA_{1}\ldots fA_{i-1},fA_{i+1\ldots .}fA_{n}. \end{array}$$

The traditional method is to estimate a maximum range for every variable and partition the range because of an equal distance with the number *n*, as well as determine the joint PDF for all instances. The PDF has, therefore, generated at an arbitrary position *A*_*i*_^*K*^ by the following equations:

(4) $$\begin{array}{c} s\left(A_{i}^{K}\right)\propto \overset{nm}{\underset{x_{1}=1}{\sum }}\ldots \overset{nm}{\underset{x_{1}-1=1}{\sum }}\overset{nm}{\underset{x_{1}+1=1}{\sum }}\ldots \overset{nm}{\underset{x_{n}=1}{\sum }}r\left(A_{1}^{x_{1}},\ldots A_{1-1}^{x_{1}-1},A_{1}^{K},A_{1+1}^{x_{1}+1}\ldots .A_{n}^{x_{n}}\right),\\ K=1,\ldots ,nm. \end{array}$$

The overall amount of PDF computations throughout this strategy is *nm*^*n*^, which also gets computationally intensive as the multitude of variables increases. To optimize performance, a simplified approach based on Latin hypercube sampling (LHS) is suggested in this study. As an example, imagine a joint PDF with two variables *A*_1_ and *A*_2_. Combine these ranges by *nm* = 8 to get 8 *∗* 8 = 64 cells, and create points by the LHS such that every column and row of the square has just one sampling. Traditionally, the quantity is produced by adding the PDF numbers at each position all along a continuous line. The number is totaled at the spots that have relocated with the same *A*_2_ from the LHS spots in the LHS approach. The motion is represented by arrows in the diagram. In this simple 2-D situation, both the traditional and LHS methods are similar, albeit taught differently. However, as demonstrated in the example of three variables, it does not apply when the variables are raised. The LHS elements are produced with an interval count of *nm*=8. To calculate the marginal PDF value at any random *A*_1_, the typical way is to add all the PDF readings at 8=64 points on the *A*_2_ − *A*_3_ planes provided by the translucent grey. Nevertheless, just for performance, only 8 points have migrated from the initial LHS points with the same *A*_2_, *A*_3_ are employed in the suggested method. The marginal PDF of parameter *A*_*i*_ by the LHS technique is provided by the expression given as follows:

(5) $$\begin{array}{c} s\left(A_{i}^{K}\right)\propto \overset{nm}{\underset{x_{1}=1}{\sum }}r\left(A_{1}^{x},\ldots A_{1-1}^{x},A_{i}^{K},A_{1+1}^{x}\ldots .A_{n}^{x}\right),\\ K=1\ldots ,nm. \end{array}$$

The *nm* calculations are at any random*A*_*i*_ that must be continued across *K* = 1,…, *nm*. For each variable *A*_*i*_, *nm*^2^ calculations will be performed and *nm*^2^ ^*∗*^*n* numbers will be determined for all the parameters, whereas the typical technique requires *nm*^2^. When these two methods are compared, the LHS technique requires significantly less calculation. Though proven with a small proportion *nm* = 8, the amount in actuality is frequently in the tens of thousands. For *n*, however, just a few values fewer than ten are generally considered. Many computational environments could improve efficiency by calculating all *nm* PDFs at any arbitrary *A*_*i*_^*K*^ in a single phase. Furthermore, in practice, the marginal PDF is not generated at each, *k* = 1,…, *nm*, which is still too expensive. Rather than *nm*, the value of every variable is separated by a considerably smaller amount *nm* as low as so many tens, but all nm PDFs were generated in a single step, as previously stated. After all, the overall amount of calculations is reduced to 1*∗nm∗n*, a far more solvable quantity in terms of processing performance.

The article "Estimation of Parameters on Probability Density Function Using Enhanced GLUE Approach" was published in 2022. Journal: Comput Intell Neurosci.

The LHS technique's marginal PDF is then used as a proposition density to create an effective and resilient GLUE procedure. Consider the following target PDF with two parameters as an example:

(6) $$\begin{array}{c} r\left(a1,a2\right)\propto \overset{4}{\underset{n=1}{\prod }}Z_{n}^{Y_{n}}{\left(1-Z_{n}\right)}^{5-Y_{n}}. \end{array}$$

Here, we get

(7) $$\begin{array}{c} \vartheta \left(\alpha |X\right)=\frac{\exp\left[a1+a2\right]}{1+\exp\left[a1+a2\right]}. \end{array}$$

### 4.3. Assessment Predicted Values and Parameter Estimations

The vectors of the subsequent average $\bar{\alpha }$ are calculated for every posterior distribution. Therefore, $\bar{\alpha }$ is taken into account as an estimation of the mathematical model vectors *α*. For every variable excepting *x*6, *y*6, and *z*6, the average absolute difference between the parametric test and the genuine parameter number is determined. Hence, the absolute deviation reflects the actual value of the parameter. Since the real values for all three factors are zero, can be simply utilized the significant differences between the estimated parameters and the real values to evaluate the predicted values of *x*6, *y*6, and *z*6.

Because the input parameter estimation techniques were frequently included to forecast *b*, it is essential to assess the reliability of model predictions whenever the parameters were set to the parameter estimates. According to [26],the model predicts *b* values by employing $\bar{\alpha }$ as parameter estimation methods. The reliability of the predicted results is then assessed by computing the mean squared error of prediction (MSEP) values. The models were employed with the real parameters in order to produce 1000 observations; the mean squared error of prediction connected with every vector $\bar{\alpha }$ is predicted in the following equation:

(8) $$\begin{array}{c} MSEP\left(\bar{\alpha }\right)=\frac{1}{1000}\overset{1000}{\underset{i=1}{\sum }}{\left[b_{i}-f\left(\beta_{i};\bar{\alpha }\right)\right]}^{2}. \end{array}$$

Assuming parameters of the model were adjusted to the posterior means, $f\left(\beta_{i};\bar{\alpha }\right)$ is the modeling prediction. For every element of *α* in the posterior parameter distribution, this is the suggested estimating value for mean squared error. MSEP's posterior distribution could then be derived.

The article "Estimation of Parameters on Probability Density Function Using Enhanced GLUE Approach" was published in 2022. Journal: Comput Intell Neurosci.

## 5. Results

### 5.1. Validation of the Enhanced GLUE Sampling Techniques

The effectiveness of the modified GLUE is demonstrated using many engineering challenges that scholars have recently researched. Because the focus is on sampling performance from the perspective of engineering applications, every topic is only briefly described. The suggested method's outcomes are determined by the standard GLUE. In all instances, the method is carried out with the amount of LHS *nm*=1000 as well as the number of GLUE iterations *n*=500. For the proposition density in traditional GLUE, a uniform distribution having finite duration is used.

#### 5.1.1. Problem with Spring

Despite finite element analysis (FEA) being a useful method for examining structure elements' fatigue performance, it frequently fails to correctly forecast the existence owing to the intrinsic unpredictability of the fatigued variables. On the contrary, practically every organization conducts live tests at the end of the development process for quality assurance (QA). As a result, the information is collected on its own. Inspired by this, a Bayesian approach is created that uses these testing data to inversely predict the fatigue-life variables. The posterior distributions of the variables are computed based on the life data acquired from the QA tests on a regular basis. The level of uncertainty in the variables might well be decreased considerably when more data are collected. A high cycle fatigue concern of a car suspension coil spring was examined throughout this relation [27]. Life is projected utilizing the stress-life relationship and the Goodman model in the following equation:

(9) $$\begin{array}{c} G={\left(\frac{R_{x}/\left(1-R_{s}/R_{ul}\right)}{y}\right)}^{1/y}. \end{array}$$

Where *x*, *y* are the stress-life coefficients, *R*_*ul*_ is the ultimate strength, while *R*_*s*_ and *R*_*x*_ are the average and alternation stresses, respectively. This happens during lifetime testing of the springs The variable *y* is considered to remain constant at −0.0725 for the sake of demonstration. The unknown variables are then *x* and *R*_*ul*_. Assume that have 9 life test results for the three different springs of the same materials stated in Table 1 that have been standardized for ease of use. The following is the posterior distribution of the uncertain variables:

(10) $$\begin{array}{c} r\left(x,R_{ul},\alpha \right)\propto \alpha^{-1}\text{exp}\left[-\frac{1}{2\alpha^{2}}\overset{9}{\underset{c=1}{\sum }}{\left.{\left(b\right.}_{c}^{e}-b_{c}^{a}\right)}^{2}\right]. \end{array}$$

The real lives acquired by the testing as well as the expected life by the FEA are denoted by *b*_*c*_^*e*^ and *b*_*c*_^*a*^, respectively. The measurement error is multiplied by the unknown variables.

The article "Estimation of Parameters on Probability Density Function Using Enhanced GLUE Approach" was published in 2022. Journal: Comput Intell Neurosci.

MCMC is used to incorporate the testing findings of the probability distribution function of the uncertain variables of enhanced GLUE. When the two outcomes are compared, the PDF forms are determined to be very similar. With the same structure, the association feature between *x* and *R*_*ul*_ is also visible. Table 1 shows the A1 and A10 life spans, which are in close proximity.  Table 2 also includes proportions and confidence intervals (C.I.) for the parameters.

However, it should be noted that the MCMC result was acquired after dozens of trials and errors with regard to the size of proposition density, which is a uniform distribution, in terms of achieving convergence. It has taken a very long time. Improved GLUE, on the other hand, achieves the same outcome in just 50 seconds in a single effort. Furthermore, as shown in the following points, MCMC is only successful in this problem with three factors, and it loses whenever there have been more than this quantity. The enhanced GLUE, on the other hand, consistently produces convergence outcomes in just a few tries, despite the number of variables.

#### 5.1.2. The Problem of Crack Growth

The framework utilizes the Paris approach to calculate damaged growth parameters depending on the calculated crack size across a number of cycles. The variables are quite often distributed widely among seemingly identical structures due to several uncertainties. The Bayesian approach is used to modify the distributions of such characteristics over time. The crack size is indicated in measures of the cycles *C* as per the Paris law shown in the following equation:

(11) $$\begin{array}{c} x\left(C\right)={\left[Cn\left(1-\frac{p}{2}\right){\left(\alpha \vartheta^{2}\right)}^{2}+x_{i}^{1-\left(p/2\right)}\right]}^{\left(2/2\right)-p}. \end{array}$$

When *n* and *p* are the 2 damage growth factors that need to be predicted, *x*_*i*_ is the expected beginning crack size, and *α* is the stress variation due to fatigue stressing. Assume it has ten large datasets of crack size measurements from a variety of cycles. Based on the preceding data of two variables, the posterior distribution of the uncertain variables is calculated as follows:

(12) $$\begin{array}{c} r\left(p,n,y,\alpha \right)\propto {\left(\frac{1}{{\left(\alpha \vartheta^{2}\right)}^{2}}\right)}^{10}\exp\left[-\frac{1}{2\alpha^{2}}\overset{10}{\underset{c=1}{\sum }}{\left(x_{mc}-x\left(C_{c}\right)-y\right)}^{2}\right]r\left(p\right)*r\left(n\right), \end{array}$$

Here,

(13) $$\begin{array}{c} r\left(p\right)=V_{\left[2,2,3,2\right]},\\ r\left(n\right)=V_{\left[\log\left[6*10^{-12}\right],\log\left[6*10^{-13}\right]\right]}. \end{array}$$

Two variables *x*and *y* are appended to the uncertainties in (12), which have been the noise and bias measurements biases, respectively. As a result, there are four unknown parameters. Synthesis data are utilized in this problem to investigate the effects of noise and bias. The actual crack diameters are calculated as per (11) for a given *C*, and the true crack data are purposefully added with a deterministic bias and random noise.

The article "Estimation of Parameters on Probability Density Function Using Enhanced GLUE Approach" was published in 2022. Journal: Comput Intell Neurosci.

These data will be used to determine the unknown variables. Despite numerous experiments, adequate sampling could not be achieved by using MCMC as depicted in Figure 1 The outcome of the improved GLUE, on the other hand, is better, and it may be reached in around two minutes with one effort.

Figure 2 depicts the enhanced GLUE measures, the produced PDF forms appear to be pretty credible, and the relationship between *p* and *n* is plainly visible. The solid blue curve represents genuine crack growth; the 90 percent prediction interval (PI) represents the red dashed line as shown in Figure 3. As predicted, MCMC failed to accurately estimate growth. The improved GLUE, on the other hand, accurately forecasts crack growth by addressing the bias and adopting the genuine model.

#### 5.1.3. The Problem of Solder Joint

The final instance is estimating the viscoplastic properties of materials of a solder junction in a microelectronics packaging in reverse. As shown in Figure 4, a solder joint experiment is developed so that the connection deforms similarly to the real packaging. Moire interferometry is used to quantify the distortion. The sample is subjected to viscoplastic FEA using the Anand model [28]. The parameters of the model are correspondingly set such that the anticipated distortion matches the experimental results during five different heating and cooling cycles.

Utilizing likelihood estimates, the approach addresses the uncertainties caused by sampling uncertainty and a lack of appropriate experimental results. Initially, the Anand concept required nine variables; however, after a sensitivity assessment, the set of parameters is decreased to the four that have the greatest influence, while the rest are left as fixed values. The posterior distribution, then again, is as follows:

(14) $$\begin{array}{c} r\left(A_{0},\frac{C}{D},X,\varepsilon ,\alpha \right)\propto {\left(\frac{1}{2\vartheta \alpha^{2}}\right)}^{15}\exp\left[-\frac{1}{2\alpha^{2}}\overset{12}{\underset{c=1}{\sum }}{\left(b_{c}^{e}-{\overset{\wedge }{b}}_{c}^{f}\right)}^{2}\right]. \end{array}$$

Here, *A*_0_, (*C*/*D*), *X*, *ε*, and *α* are Anand parameters and systematic errors were applied according to the evaluated value. *b*^*e*^. and ${\overset{\wedge }{b}}^{f}$ in the equations represent the solder movement acquired by experimental and analytical models, respectively. The cap symbol in ${\overset{\wedge }{b}}^{f}$ signifies the responsive surface model, which is provided by second-order polynomials in terms of the following 4 parameters to substitute the time-consuming FEA. The sample is put through the temperature cycle shown in Figure 4.

The article "Estimation of Parameters on Probability Density Function Using Enhanced GLUE Approach" was published in 2022. Journal: Comput Intell Neurosci.

The PDFs and the sampled outcomes of the uncertain variables were generated using the enhanced GLUE. Also identified are the connections among *A*_0_ and (*C*/*D*), as well as *ε* and *X*. Although the presence of two pairs of intricate connections between the variables could affect sample drawing challenges, the findings are produced in around eight minutes [29].

The MCMC solution for this issue could never be produced at all.  Figure 5 shows the posterior predictive distributions of movement produced from the sampling data. The blue line containing diagonal marks in the pictures represents the MCMC experimental outcomes. The red line containing the square represents the average of the predictive distribution derived by the enhanced GLUE [30].

Figure 6 shows the posterior predictive distributions of pressure produced from the sampling data. At every occurrence, the 90 percent prediction boundaries are also represented utilizing vertical lines. The results of the FEA based on the existing literature are significantly varied from the experimental data, as seen in the figures. The average of the anticipated distributions gets significantly closer to the experimental values following inversely predicting the properties of materials [31].

### 5.2. Estimation of MSEP

Considering 1000 or 2000 generated parameter sets, two alternative beginning values, and 5 or 40 data samples, the posterior averages were calculated using the MCMC and GLUE methods.  Table 3 illustrates the MSEP results calculated by fixing the parameters of the model to the posterior means. The performance was acquired for 100 samples of data, not for one specific sample of data points *X*. The vectors of the posterior variable distribution's averages$\bar{\alpha }$ were calculated for every sample by using the GLUE technique [32]. (8) was then used to determine the MSEP value assigned to every $\bar{\alpha }$ value. Lastly, the individual MSEP results were used to estimate the MSEP's predicted values over the 100 data samples.

The article "Estimation of Parameters on Probability Density Function Using Enhanced GLUE Approach" was published in 2022. Journal: Comput Intell Neurosci.

The MSEP of the models is 17.17 once the requirements are identified to their preceding means. That value is significantly greater than the remaining error variance *α*^2^, which is equivalent to 0.16 and indicates the model's smallest possible MSEP, so that it is the MSEP with the actual attribute values. Because when estimated values are set to the averages of the posterior parameter distribution obtained utilizing MCMC or the GLUE technique, the MSEP is significantly reduced. The MCMC and 2000 iterations get the least MSEP value (0.21). This result is quite close to the minimum MSEP value, which is 0.16. The MSEP has no meaningful effect on the beginning values. Once six data samples have been used, the computational time has a minor impact on the MSEP value, however, when fifty data samples are used, which has no impact. The Bayesian approach used to construct the posterior parameter distributions has little effect on the MSEP value. Whenever the number of data samples is 50, the predicted MSEP values produced using the GLUE approach are marginally greater [33]. The prior parameter distribution, on the other hand, has a significant impact on MSEP values. The anticipated MSEP results calculated with 6 and 50 data samples are 5.67 and 1.86, respectively, whenever the previous distribution having reduced variations is employed. Such MSEP is significantly greater than the actual preceding distribution values. That's because the true values of parameters are not included in the parameter space represented by the prior distribution having lower variations. As a result, even when a large set of data sets are employed, the posterior means of such variables generally remain distinct from the genuine parameter values.

## 6. Conclusion

Parameter estimation of probability density functions is one of the most significant processes in statistical image and signal processing (PDF). In the fields of artificial intelligence and machine learning, estimating the probability density function is a contentious topic. The research focuses on difficulties in estimating a density function from its random variable. When only minimal density forecasts are given, the paper presents a framework for evaluating probability density functions. Sampling is commonly used to estimate and describe the probabilistic model of unknown variables in the Bayesian approach, which is to provide correct samplings that reflect the probability aspect of the variables. The generalized likelihood uncertainty estimation (GLUE) approach has gained the most popular among the numerous methodologies due to its efficacy and wide application. The Bayesian method allows model parameters to be calculated based on prior knowledge of parameter outcomes and experimental observations. To address these difficulties, the investigation offers a strategy that employs the marginal probability density function (PDF) as a distribution to demonstrate the utility of the proposed method; specific engineering problems created using the Bayesian methodology are addressed. Despite this, the model's mean squared error of prediction is significantly larger when employing the GLUE technique than with the preceding algorithms. The results of the approaches are influenced by the assumptions made about parameter values in advance. The ideas of learning and prediction accuracy are discussed, as well as the value of a statistical experiment. These ideas are useful to demonstrate that the GLUE technique defines an incomplete statistical inference process. Despite the fact that numerous sampling techniques have been created, there is not a reliable, affordable solution that could address real-world issues in an engineering application. The most successful sampling technique, known as GLUE, has the drawback of becoming ineffective as the amount of parameters rises and the values become more closely connected. Prior to the primary GLUE technique, this method requires additional computation for marginal PDF creation. Instead, better resilience and efficiency are attained by such an approach since it always obtains convergent samples, that is, the identical samples when the technique is applied that were not achievable while using MCMC. In summary, a very useful technique to handle parameter estimation in the scenario of higher parameters as well as correlations is the GLUE combined with the marginal distribution, which is discussed. The numerous real-world engineering issues where sufficient samples are gathered for the posterior distribution serve as evidence for the method's viability.

The article "Estimation of Parameters on Probability Density Function Using Enhanced GLUE Approach" was published in 2022. Journal: Comput Intell Neurosci.

## Figures and Tables

**Figure 1:** MCMC growth of crack estimation.

**Figure 2:** GLUE growth of crack estimation.

**Figure 3:** Solder joint sample.

**Figure 4:** Temperature cycle.

**Figure 5:** Preceding estimation of movement.

**Figure 6:** Preceding estimation of pressure.

**Table 1:** Testing surveillance of spring and estimated A1 and A10.

	Data testing			Estimated surveillance		
	1-Real surveillance	2-Real surveillance	3-Real surveillance	A1	A10	Techniques
1^st^ type of spring	0.0327	1.7745	1.3124	1.2198	1.6277	MCMC
				1.1311	1.2585	GLUE

2^nd^ type of spring	15.2246	8.8312	4.2734	6.1225	8.1337	MCMC
				4.0244	6.1157	GLUE

3^rd^ type of spring	1.1780	1.1007	1.1845	1.1548	1.1812	MCMC
				1.1321	1.1514	GLUE

**Table 2:** Proportions and CI of variables.

Variables	Techniques	Proportion			
		*r*-10th	Average	*r*-90th	Confidence interval-95th
*x*	MCMC	2.2171	2.1418	2.2614	0.3511
	GLUE	1.2783	2.0598	2.2176	0.2869

*R*_*ul*_	MCMC	1.7623	2.4355	2.1787	0.1752
	GLUE	1.3824	2.1245	2.0472	0.0638

*α*	MCMC	0.1083	0.1156	0.4932	0.1141
	GLUE	0.0769	0.1722	0.2346	0.1581

**Table 3:** MSEP prediction analysis.

Amount of data	Techniques	Amount of iterations	Initial parameters	$\hat{e}\left(\text{MSEP}\left(\bar{\alpha }\right)\right)$
*Beginning of the preceding parameter distribution*				
0	—	—	—	15.32
6	MCMC	1000	2	4.91 (1.3)
6	GLUE	1000	—	2.52 (0.31)
6	MCMC	2000	1	3.72 (0.56)
6	GLUE	2000	—	4.21 (0.28)
50	MCMC	1000	2	1.33 (0.5)
50	GLUE	1000	—	1.33 (0.33)
50	MCMC	2000	2	1.17 (0.52)
50	GLUE	2000	—	1.20 (0.06)

*Preceding parameters having lower variations*				
6	MCMC	1000	2	4.53 (1.23)
50	MCMC	1000	2	2.92 (0.03)

## Data Availability

The data used to support the findings of this study are available from the corresponding author upon request.
